The article "Fibulin-5 inhibits hepatocellular carcinoma cell migration and invasion by down-regulating matrix metalloproteinase-7 expression" was retracted in 2025. Reasons: duplicated images; overlap with earlier publications; unreliable data; concerns about the images.

# Fibulin-5 inhibits hepatocellular carcinoma cell migration and invasion by down-regulating matrix metalloproteinase-7 expression

**DOI:** 10.1186/1471-2407-14-938

**Published:** 2014-12-12

**Authors:** Kangsheng Tu, Changwei Dou, Xin Zheng, Chao Li, Wei Yang, Yingmin Yao, Qingguang Liu

**Affiliations:** Department of Hepatobiliary Surgery, the First Affiliated Hospital of Xi’an Jiaotong University, Xi’an, 710061 PR China

**Keywords:** Fibulin-5, Hepatocellular carcinoma, Migration, Invasion, MMP-7

## Abstract

**Background:**

Fibulin-5 has been considered as a tumor suppressor through inhibiting tumor growth and invasion. Reduced expression of Fibulin-5 is frequently observed in various human cancers. In this study, we investigate the clinical significance of Fibulin-5 and its role in hepatocellular carcinoma (HCC) cell migration and invasion.

**Methods:**

The expression of Fibulin-5 was evaluated by qRT-PCR and immunoblotting in HCC and matched noncancerous tissues. Fibulin-5 was over-expressed or knocked down by a retrovirus-mediated expression plasmid or a specific siRNA in HCC cells. Boyden chamber and Transwell assays were used to test HCC cell migration and invasion. Immunostaining was performed to determine matrix metalloproteinase-7 (MMP-7) expression in HCC specimens. MMP-7 retroviruses and siRNA were used to alter MMP-7 expression in HCC cells.

**Results:**

In our study, the expression levels of Fibulin-5 protein and mRNA were down-regulated in HCC tissues as compared with those in matched noncancerous tissues. Reduced expression of Fibulin-5 was observed in all HCC cell lines (HepG2, SMMC-7721, MHCC97L, Hep3B, MHCC97H and HCC-LM3) as compare with that in a non-transformed hepatic cell line (LO2). Low expression of Fibulin-5 was significantly correlated with poor prognostic features including multiple tumor nodes, venous infiltration, high Edmondson-Steiner grading and advanced tumor-node-metastasis (TNM) tumor stage. Furthermore, we demonstrated that Fibulin-5 was a novel independent prognostic marker for predicting 5-year survival of HCC patients. Our *in vitro* studies showed that Fibulin-5 overexpression inhibited HCC cell migration and invasion. While Fibulin-5 knockdown increased the number of migrated and invaded HCC cells. Fibulin-5 negatively regulated MMP-7 abundance in HCC cells. Moreover, the inverse correlation between Fibulin-5 and MMP-7 expressions was observed in HCC tissues. Mechanistically, we disclosed that MMP-7 knockdown reduced the number of migrated and invaded HCC cells. Restoring MMP-7 expression abrogated the suppressive effect of Fibulin-5 on HCC cell migration and invasion *in vitro*, suggesting that Fibulin-5 exerted its anti-metastatic function, at least in part, by down-regulating the expression of MMP-7 in HCC cells.

**Conclusions:**

These results indicate that Fibulin-5 may serve as a prognostic biomarker and inhibits HCC invasion and metastasis by suppressing MMP-7 expression.

## Background

Fibulin-5 is a member of Fibulin family, which are characterized by calcium-binding epidermal growth factor (EGF)-like repeats and a globular carboxyl-terminal Fibulin type structure [1, 2]. Distinct from other members, Fibulin-5 contains an integrin-binding RGD motif which binds to integrins and mediates endothelial cell adhesion [3, 4]. Functionally, Fibulin-5 is involved in cell-to-cell and cell-to-matrix communication; it also regulates the extracellular matrix structure and functions in fibrogenesis, angiogenesis and tumorigenesis [5–7].

Fibulin-5 expression was down-regulated in the malignancies of kidney [8], breast [9], ovary [9], colon [9], prostate [10], bladder [11] and lung [12]. *In vitro* studies showed Fibulin-5 inhibited proliferation and invasion of human bladder cancer cell [11]. In melanoma, histamine promoted tumor growth partly through suppressing Fibulin-5 expression [13]. Fibulin-5 has also been implicated in inhibiting lung cancer metastasis by modulating matrix metalloproteinase7 (MMP7) expression [12]. These studies indicate that Fibulin-5 probably functions as a suppressor for tumor formation and metastasis. However, other studies showed the pro-tumor role of Fibulin-5. Fibulin-5 was found to enhance the malignancy of human fibrosacroma cells [9]. Fibulin-5 expression was found to be stimulated by transforming growth factor (TGF)-beta in mammary epithelial cells (MECs) and its upregulation resulted in MEC invasion and epithelial-mesenchymal transition (EMT) via a MMP-dependent mechanism [14]. Oncogenic Fibulin-5 promotes nasopharyngeal carcinoma cell metastasis correlates with poor prognosis [15]. In Hela cells that overexpress Nogo-B, cell migration and invasion was promoted by the elevated secretion of Fibulin-5 [16]. Therefore, the precise function of Fibulin-5 in tumorigenesis and metastasis varies between different cancer types. However, Fibulin-5 in the initiation and progression of HCC remains poorly understood.

In this study, we find that Fibulin5 expression is impaired in HCC. Clinical analysis indicates that Fibulin-5 has a prognostic role in predicting survival of HCC patients. Fibulin-5 inhibits cell migration and invasion and inversely regulates MMP-7 abundance in HCC cells. Importantly, the anti-metastatic effect of Fibulin-5 is inverted by restoring MMP-7 expression *in vitro*. Our results suggest that Fibulin-5 may inhibit MMP-7 expression, thereby suppressing HCC metastasis and hence tumor progression.

## Methods

### Clinical samples

86 HCC samples were collected from patients including 69 males and 17 females, who underwent the resection of their primary HCC in the Department of Hepatobiliary Surgery at the First Affiliated Hospital of Xi’an Jiaotong University during January 2006 to December 2008. Patients did not receive preoperative chemotherapy or embolization. All samples were used after obtaining informed consent. The demographic features and clinicopathologic date are shown in Table 1. The Xi’an Jiaotong University Ethics Committee approved all protocols according to the Declaration of Helsinki (as revised in Tokyo 2004).

**Table 1:** **Clinical correlation of Fibulin-5 expression in HCC**

Clinicopathologic features		Total No. of patients, n = 86	No. of patients		*P*
			Fibulin-5 ^low^	Fibulin-5 ^high^	
Age (y)	<50	27	15	12	0.208
	≥50	59	41	18	
Sex	Male	69	44	25	0.597
	Female	17	12	5	
HBV	Absent	30	19	11	0.800
	Present	56	37	19	
Serum AFP level (ng/mL)	<400	34	24	10	0.389
	≥400	52	32	20	
Tumor size (cm)	<5	30	22	8	0.242
	≥5	56	34	22	
No. of tumor nodules	1	66	49	17	0.001*
	≥2	20	7	13	
Cirrhosis	Absent	37	26	11	0.384
	Present	49	30	19	
Venous infiltration	Absent	42	33	9	0.011*
	Present	44	23	21	
Edmondson-Steiner grading	I + II	29	24	5	0.014*
	III + IV	57	32	25	
TNM tumor stage	I + II	61	44	17	0.033*
	III + IV	25	12	13	

HCC, hepatocellular carcinoma; HBV, hepatitis B virus; AFP, alpha-fetoprotein; TNM, tumor-node-metastasis. *Statistically significant.

### Western blot

Fibulin-5 (R&D system, Minneapolis, MN, USA) and MMP-7 (EMD BioSciences, San Diego, CA, USA) and GAPDH (G8140, US Biological, Salem, MA, USA) antibodies were used for immunoblotting assay as previously described [17].

### Real-time quantitative reverse transcription polymerase chain reaction (qRT-PCR)

Fibulin-5 primers (forward: 5′-TCGCTATGGTTACTGCCAGCA-3′; reverse: 5′-TTGGCAAGACCTTCCATCGTC-3′). The PCR amplification for the quantification of the Fibulin-5 mRNA and the GAPDH mRNA was performed using a SYBR® Premix Ex Taq™ ii (Perfect Real Time) Kit (Takara Bio, Shiga, Japan), as previously described [18].

### Immunohistochemical staining

Immunohistochemistry was performed with mouse antibodies against Fibulin-5 (R&D system) and MMP-7 (EMD BioSciences) as previously described [19]. The percentage of positive tumor cells was graded as per the following criteria: 0, less than 10%; 1, 10–30%; 2, 31–50%; 3, more than 50%.

### Cell lines and transfection

The human immortalized normal hepatocyte cell line, LO2, and six HCC cell lines, HepG2, MHCC97L, Hep3B, SMMC-7721, MHCC97H and HCC-LM3 (the Institute of Biochemistry and Cell Biology, Chinese Academy of Sciences, Shanghai, China), were cultured in complete Dulbecco’s modified Eagle medium (DMEM, Gibco, Grand Island, NY, USA) containing 10% fetal bovine serum (FBS, Gibco) with 100 units/mL penicillin and 100 μg/mL streptomycin (Sigma, St-Louis, MO, USA) in a humidified containing of 5% CO2 incubator at 37°C.

Retroviral vectors pMMP-Fibulin-5 and pMMP-MMP-7 were generated by inserting the cDNA into pMMP. Retrovirus packaging and transduction were described previously [20]. Fibulin-5 was knocked down using a small interfering RNA (siRNA) duplexes (ON-TARGETplus siRNA J-017621-05 and -06; GE Dharmacon, Chicago, IL, USA). MMP-7 was knocked down by *MMP-7 757* (GGCAUUCAGAAACUAUAUG) and *MMP-7 877* (GCACUGUUCCUCCACUCCA) (GE Dharmacon) [12]. Cells were transfected with the siRNAs mentioned above using Lipofectamine 2000 according to the manufacturer’s instructions (Invitrogen, Carlsbad, CA, USA).

### Boyden chamber and Transwell assays

A Boyden chamber assay (NeuroProbe, Gaithersburg, MD, USA) was used to analyze HCC cell migration as previously described [21]. Transwell assays were done in 6 well plates with Transwell inserts equipped with 8-μm pores (Nalge Nunc International Corp, Naperville, IL, USA) coated with Matrigel at 1:6 dilution (Becton Dickinson Labware, Bedford, MA, USA) as previously described [22].

### Statistical analysis

Results are expressed as Mean ± SEM. Significance was established, with the SPSS statistical package for Windows Version 13 (SPSS, Chicago, IL, USA) and GraphPad Prism 5 software (GraphPad Software, Inc, San Diego, CA, USA), using a Pearson chi-squared test, the multi-variant Cox regression analysis, a two-tailed Student’s t test, a Kaplan–Meier plot, a log-rank test, a Spearman’s rank correlation coefficient or an ANOVA when appropriate. Difference were considered significant when *P* < 0.05.

## Results

### The expression of Fibulin-5 in HCC specimens and cells

Initially, we tested Fibulin-5 expression in a retrospective cohort of 86 HCC samples using Western blot. In these cases, we found that Fibulin-5 expression in HCC tissues was prominently lower than that in matched tumor-adjacent tissues (*P* < 0.05, Figure 1A). 20 pairs of tumor tissues and matched adjacent nontumor tissues were subjected to qRT-PCR for Fibulin-5 mRNA. The difference of Fibulin-5 mRNA levels between cancer and noncancerous tissues were the same as protein levels (tumor: 0.92 ± 0.10 *vs* nontumor: 1.93 ± 0.12, *P* < 0.05). Furthermore, Fibulin-5 mRNA levels were down-regulated in HCC cell lines, Hep3B, HepG2, MHCC97L, SMMC-7721, MHCC97H and HCC-LM3, as compared with that in normal hepatocyte cell line, LO2 (*P* < 0.05, Figure 1B). Moreover, Fibulin-5 expression in the highly metastatic HCC cell lines, MHCC97H and HCC-LM3, were obviously lower than those in the low metastatic HCC cell lines including HepG2, MHCC97L, SMMC-7721 and Hep3B (*P* < 0.05, Figure 1B). As determined by Western blot, the levels of Fibulin-5 protein showed the same pattern as mRNA levels in all cell lines (Figure 1B). Thus, our data indicate that Fibulin-5 is down-regulated in HCC tissues and cells.

**Figure 1:** **Expression of Fibulin-5 in HCC. A)** Representative Western blot analysis of Fibulin-5 expression in the HCC (T) and matched adjacent nontumor tissues (NT) was shown. Quantification of the data revealed that Fibulin-5 protein expression level in the cancer tissues was significantly lower than that in the noncancerous tissues. n = 86; *P < 0.05 by t test. **B)** Comparing differences in the expression levels of Fibulin-5 between HCC cell lines with different metastatic potentials and the immortalized hepatic cell line LO2. n = three repeats with similar results; *P < 0.05 by ANOVA.

### Clinical significance of Fibulin-5 expression in HCC

We determined 0.31 as a cutoff value, which was defined as the mean of the cohort, for Fibulin-5 protein level. Fibulin-5 expression was considered as either low (<0.31, n = 56) or high (≥0.31, n = 30). As shown in Table 1, low expression of Fibulin-5 protein was prominently associated with multiple tumor nodes (*P* = 0.001), venous infiltration (*P* = 0.011), high Edmondson-Steiner grading (*P* = 0.014) and advanced tumor-node-metastasis (TNM) tumor stage (*P* = 0.033). Thus, our results indicate that the reduced expression of Fibulin-5 is correlated with poor prognostic features of HCC. Next, 86 HCC patients with clinical survival information (with a median follow-up time of 35.5 months) were analyzed by Kaplan Meier estimation. Tumors with high expression of Fibulin-5 indeed associated with better overall survival and disease-free survival of HCC patients (*P* < 0.05, respectively, Figure 2). Furthermore, Fibulin-5 expression was an independent factor for predicting both 5-year overall and disease-free survival in HCC patients (*P* = 0.005 and 0.001, respectively, Table 2). These data indicate that Fibulin-5 may act as a potent biomarker for predicting prognosis of HCC patients.

**Figure 2:** **Prognostic significance of Fibulin-5 in HCC cases.** Kaplan-Meier 5-year **A)** overall and **B)** disease-free survival curves of HCC patients according to the level of Fibulin-5 protein expression. The Fibulin-5 high expression group (>0.31, n = 30); Fibulin-5 low expression group (<0.31, n = 56). The mean expression value obtained for Fibulin-5 of the 86 HCC samples detected by Western blot was chosen as the cutoff value. *P < 0.05 by log-rank test.

**Table 2:** **Multivariate Cox regression analysis of 5-year overall and disease-free survival of 86 HCC patients**

Variables	Overall survival			Disease-free survival		
	HR	95% CI	*P*	HR	95% CI	*P*
No. of tumor nodules	1.701	0.666-4.342	0.267	1.064	0.209-5.421	0.940
Venous infiltration	1.054	0.999-1.112	0.056	1.067	0.504-2.260	0.865
Edmondson-Steiner grading	2.230	0.937-5.308	0.070	1.971	0.827-4.696	0.126
TNM tumor stage	1.023	1.002-1.044	0.032*	1.055	1.019-1.092	0.003*
Fibulin-5 expression in tumor	2.148	1.255-3.677	0.005*	3.547	1.644-7.653	0.001*

TNM, tumor-node-metastasis; HR, hazard ratio; CI, confidence interval. *Statistically significant.

### Fibulin-5 inhibits HCC cell migration and invasion

We transduced HCC cell line, HCC-LM3, with empty vector (EV) or Fibulin-5 retroviruses. As measured by Western blot, the level of Fibulin-5 protein was significantly up-regulated by ectopically expressing Fibulin-5 in HCC-LM3 cells (*P* < 0.05, Figure 3A). Boyden chamber assays were performed to test the effect of altering Fibulin-5 levels on HCC cell migration. We found that Fibulin-5 overexpression led to a significant reduction of cell migration in HCC-LM3 cells (*P* < 0.05, Figure 3B). Furthermore, as determined by Transwell assays, the number of invaded HCC-LM3 cells was significantly reduced after Fibulin-5 overexpression (*P* < 0.05, Figure 3B). Next, Fibulin-5 was knocked down by a specific siRNA in MHCC97L cells (*P* < 0.05, Figure 3C). As expected, Fibulin-5 knockdown obviously promoted HCC cell migration and invasion (*P* < 0.05, respectively, Figure 3D). However, Fibulin-5 overexpression did not significantly affect cell growth (EV: 102.20 ± 3.36 *vs* Fibulin-5: 95.00 ± 3.10, *P* = 0.148) and apoptosis (EV: %11.17 ± 1.08 *vs* Fibulin-5: %13.25 ± 1.05, *P* = 0.196) in HCC-LM3 cells. Thus, Fibulin-5 may exert an anti-metastatic effect on HCC.

**Figure 3:** **Fibulin-5 reduces HCC cell migration and invasion. A)** HCC-LM3 cells that were transfected with empty vector (EV) or Fibulin-5 retroviruses were subjected to western blot for Fibulin-5. n = six independent experiments; *P < 0.05 by *t* test. **B)** Cell migration and invasion as measured by Boyden chamber and Transwell assays were inhibited by Fibulin-5 overexpression in HCC-LM3 cells as compared with control cells. n = three repeats with similar results, *P < 0.05 by t test. HPF: high power field. **C)** MHCC97L cells that were transfected with scrambled siRNA or Fibulin-5 siRNA were subjected to western blot for Fibulin-5. n = six independent experiments; *P < 0.05 by *t* test. **D)** Fibulin-5 knockdown MHCC97L cells conferred a less number of migrated and invaded cells as compared with control cells. n = three repeats with similar results; *P < 0.05 by *t* test. HPF: high power field.

### Fibulin-5 inversely regulates MMP-7 in HCC

The inverse correlation between Fibulin-5 and MMP-7 expression was reported previously in lung cancer [12]. HCC-LM3 cells that were transfected with EV or Fibulin-5 were subjected to immunoblotting for MMP-7 protein. Interestingly, we found that Fibulin-5 overexpression significantly decreased the level of MMP-7 protein (*P* < 0.05, Figure 4A). Furthermore, Fibulin-5 knockdown obviously increased the level of MMP-7 protein in MHCC97L cells (*P* < 0.05, Figure 4B). We next detected Fibulin-5 and MMP-7 expression using immunostaining in a cohort of 86 HCC samples. Fibulin-5 or MMP-7 immunoreactivity was considered as either negative (score 0) or positive (scores 1 to 3). In these cases, MMP-7 expression was detected in 48.5% (32/66) of the HCC samples with negative Fibulin-5 expression, whereas only 15.0% (3/20) of the HCC specimens with positive Fibulin-5 expression showed a positive MMP-7 signal (*P* < 0.05, Figure 4C and 4D). Furthermore, Spearman correlation analysis indicated that Fibulin-5 was inversely correlated with MMP7 expression in HCC tissues (*r* = -0.632, *P* < 0.001). These data indicate that Fibulin-5 reduces MMP-7 protein levels in HCC.

**Figure 4:** **Fibulin-5 regulates MMP-7 abundance in HCC. A)** Fibulin-5 overexpression decreased the level of MMP-7 protein in HCC-LM3 cells. n = six independent experiments; *P < 0.05 by *t* test. **B)** Fibulin-5 knockdown led to accumulation of MMP-7 protein in MHCC97L cells. n = six independent experiments; *P < 0.05 by *t* test. **C)** In cases of high Fibulin-5 protein expression (I), there was no detectable MMP-7 protein expression (II) in the same tissue section. In contrast, in the case of low Fibulin-5 protein expression (III), there was strong MMP-7 protein expression (IV). Scale bar: 100 μm. **D)** Fibulin-5 and MMP-7 expression in 86 HCC samples analyzed by immunohistochemistry. A significant inverse correlation between Fibulin-5 and MMP-7 expression was observed in HCC. *P* < 0.05 by two-tailed chi-square test.

### Fibulin-5 inhibits HCC cell migration and invasion by suppressing MMP-7

To determine whether the MMP-7 protein participates in Fibulin-5 mediated suppression of HCC cell migration and invasion, MMP-7 expression was obviously knocked down by a specific siRNA in HCC-LM3 cells (*P* < 0.05, Figure 5A). As shown in Figure 5B, MMP-7 knockdown significantly inhibited HCC cell migration and invasion (*P* < 0.05, respectively). Furthermore, Fibulin-5 overexpressing HCC-LM3 cells were subsequently transfected with EV or MMP-7 retroviruses. Restoring MMP-7 expression in HCC-LM3 cells abolished the effect of exogenous Fibulin-5 overexpression, leading to a significant increase in the number of migrated and invaded cells (*P* < 0.05, respectively, Figure 5C and 5D). Taken together, these data indicate that MMP-7 may function as a downstream factor in Fibulin-5 mediated suppression of HCC cell migration and invasion

**Figure 5:** **Fibulin-5 exerts anti-metastatic effect by suppressing MMP-7 expression. A)** The expression of MMP-7 was knocked down by a specific siRNA in HCC-LM3 cells. n = six independent experiments; *P < 0.05 by *t* test. **B)** Boyden chamber and Transwell assays indicated that MMP-7 knockdown inhibited migration and invasion of HCC-LM3 cells. n = three repeats with similar results, *P < 0.05 by t test. **C)** Fibulin-5-expressing HCC-LM3 cells that were transfected with empty vector (EV) or MMP-7 retroviruses were subjected to immunoblotting for MMP-7. n = six independent experiments; *P < 0.05 by *t* test. **D)** Restoring MMP-7 expression increased migration and invasion in Fibulin-5 expressing HCC-LM3 cells. n = three repeats with similar results, *P < 0.05 by t test.

## Discussion

In our study, we initially detected Fibulin-5 expression status in 86 samples of surgical resected HCC tissues. Our data indicated that the level of Fibulin-5 expression in HCC was significantly lower than that in normal tumor-adjacent tissues. Reduced expression levels of Fibulin-5 mRNA were observed in HCC cell lines, especially in the highly metastatic cell lines. Furthermore, Fibulin-5 protein was expressed at significantly lower levels in HCC patients with multiple tumor nodes, venous infiltration, high Edmondson-Steiner grading and advanced TNM tumor stage. These results suggest that the reduced expression of Fibulin-5 is correlated with poor prognostic features in HCC. Importantly, our data demonstrated that high expression of Fibulin-5 was correlated with a significant better 5-year survival for HCC patients. Multivariate Cox repression analysis indicated that Fibulin-5 was an independent prognostic factor for predicting survival of HCC patients. Altogether, these results suggest that Fibulin-5 expression is critical for prognosis determination in HCC patients.

Several studies have identified Fibulin-5 as a driving tumor suppressor in human cancers [8–12]. Mechanistically, Fibulin-5 exerts anti-cancer functions by inhibiting tumor growth and metastasis [1]. In our study, we found that Fibulin-5 overexpression significantly reduced the number of migrated and invaded HCC-LM3 cells and Fibulin-5 knockdown prominently promoted MHCC97L cell migration and invasion. However, Fibulin-5 overexpression did not obviously affect cell growth and apoptosis. These data confirm that Fibulin-5 indeed inhibits HCC cell migration and invasion, not kills cells or makes cells sick. The inverse correlation between Fibulin-5 and MMP-7 expression has been reported previously and Fibulin-5 suppresses lung cancer invasion by inhibiting MMP-7 expression [12]. Our *in vitro* studies demonstrated that Fibulin-5 overexpression down-regulated MMP-7 protein in HCC-LM3 cells and Fibulin-5 knockdown led to MMP-7 protein accumulation in MHCC97L cells. Moreover, we found that the MMP-7 expression level in HCC tissues from negative Fibulin-5 expression group was prominently higher as compared with that in HCC tissues from positive Fibulin-5 expression group. Spearman correlation analysis indicated an inverse correlation between Fibulin-5 and MMP7 expression in HCC tissues. Thus, our results indicate that Fibulin-5 inversely regulate MMP-7 abundance in HCC. We further confirmed that MMP-7 knockdown by a specific siRNA inhibited HCC-LM3 cell migration and invasion, which was consistent with previous reports [23]. Furthermore, the suppression in HCC cell migration and invasion by Fibulin-5 overexpression could be reverted by restoring MMP-7 expression. Taken together, these data suggest that Fibulin-5 suppresses HCC cell migration and invasion by inhibiting MMP-7 expression. In lung cancer, suppression of MMP-7 expression by Fibulin-5 was mediated by an integrin-binding RGD motif via the extracellular signal-regulated kinase (ERK) pathway [12]. Therefore, further investigation is required to confirm the precise molecular mechanisms between Fibulin-5 and MMP-7 in HCC.

In conclusion, we find that Fibulin-5 is down-regulated in HCC and its low expression is related to malignant clinicopathologic characteristics. Moreover, Fibulin-5 expression is an independent prognostic marker for predicting 5-year survival of HCC patients. *In vitro* studies demonstrate that Fibulin-5 reduces HCC cell migration and invasion. Mechanistically, we suggest that Fibulin-5 may inhibit HCC invasion and metastasis by suppressing MMP-7. Taken together, we consider that Fibulin-5 may potentially act as a clinical biomarker, and may also be a therapeutic target, in HCC.

## Conclusions

In summary, this study shows that Fibulin-5 expression is down-regulated in tumor tissues as compared with matched adjacent nontumor liver tissues and that the low expression of Fibulin-5 confers poor prognostic features of HCC. Furthermore, we find that Fibulin-5 functions as an independent factor for predicting the 5-year overall survival and disease-free survival of HCC patients. Functional studies demonstrate that Fibulin-5 inhibits HCC cell migration and invasion. Interestingly, our data indicate that Fibulin-5 inversely regulates the abundance of MMP-7 protein in HCC cells. An inverse correlation between Fibulin-5 and MMP-7 is observed in HCC tissues. Importantly, MMP-7 knockdown suppresses HCC cell migration and invasion. Restoring MMP-7 can abolish the effect of Fibulin-5 overexpression on anti-metastasis in HCC, suggesting that Fibulin-5 may function as a metastasis-suppressor gene by downregulating MMP-7. This study reveals that Fibulin-5 may be a potential prognostic biomarker of HCC. Fibulin-5 may play a critical role in the invasion and metastasis of HCC.

## Abbreviations

HCC: Hepatocellular carcinoma
qRT-PCR: Real-time quantitative reverse transcription polymerase chain reaction
EGF: Epidermal growth factor
MMP-7: Matrix metalloproteinase-7
TGF-beta: Transforming growth factor-beta
MECs: Mammary epithelial cells
EMT: Epithelial-mesenchymal transition
FBS: Fetal bovine serum
DMEM: Dulbecco’s modified Eagle medium
ERK: Extracellular signal-regulated kinase
TNM: Tumor-node-metastasis.
